The article "Surgical Treatment and Prognosis of Angiosarcoma of the Scalp: A Retrospective Analysis of 14 Patients in a Single Institution" was published in 2015. Journal: Biomed Res Int.

# Surgical Treatment and Prognosis of Angiosarcoma of the Scalp: A Retrospective Analysis of 14 Patients in a Single Institution

**DOI:** 10.1155/2015/321896

**Published:** 2015-12-02

**Authors:** Jun Ho Choi, Kyung Chan Ahn, Hak Chang, Kyung Won Minn, Ung Sik Jin, Byung Jun Kim

**Affiliations:** Department of Plastic and Reconstructive Surgery, Seoul National University Hospital, Seoul National University College of Medicine, 101 Daehak-ro, Jongno-gu, Seoul 110-744, Republic of Korea

## Abstract

*Objective*. We describe specific surgical methods for angiosarcoma regarding extent of resection and reconstructive options and assess their effect on patients' prognosis.* Patients and Methods*. We retrospectively examined 14 patients undergoing treatment for angiosarcoma of the scalp at our institute between January 2000 and June 2015. Surgical treatment comprised wide excision of the tumor and reconstruction using a free flap with skin graft. Kaplan-Meier survival analysis was used to assess the survival parameters. Univariate and multivariate analyses were performed to evaluate the association between risk factors and outcome parameters.* Results*. Mean patient age at diagnosis was 69 years, and the mean follow-up period was 17 months. The overall 5- and 2-year survival rates were 15% and 75%, respectively, whereas the 5- and 2-year disease-free survival rates were 7.7% and 38.7%, respectively. The mean survival duration was 32 months. Metastatic tumor dissemination to the lung or brain was closely associated with the major cause of death. Only a deep excision margin was significantly related to the recurrence rate.* Conclusions*. Cases of angiosarcoma had a poor prognosis despite the aggressive treatments. Sufficient resection margins are essential for controlling local recurrence. The effect of multidisciplinary approaches needs to be explored.

## 1. Introduction 

Angiosarcoma (AS) is rare vascular neoplasm affecting the endothelial cells of blood vessel. Cutaneous AS usually develops in the face or scalp [1, 2]. This tumor predominantly develops in elderly people and more frequently affects men than women [2–4]. AS accounts for less than 2% of all cases of soft-tissue sarcoma and less than 1% of cases of head and neck cancer [5–7]. The etiology of AS has not been fully understood, but several reports have shown some positive association with chronic lymphedema [8] or prior irradiation [9, 10]. It is a highly aggressive malignant tumor with a high rate of locoregional recurrence and tends to metastasize at an earlier stage. Although various active treatment options have been adopted, the associated prognosis remains poor. Many studies have indicated that the 5-year survival rate of AS ranges between 10% and 50% [4, 7, 11–13]. No common consensus has been reached regarding the optimal treatment [6]. However, a multimodality approach of wide excision and radiotherapy is broadly accepted as the standard treatment [2, 6, 14]. As concrete surgical strategies have still not been established, in the present report, we describe surgical methods for AS in terms of the extent of resection and reconstructive options and assess their effect on patient prognosis.

## 2. Materials and Methods

### 2.1. Study Design and Patients

The subjects of the present study are patients with AS of the scalp, who were treated at our institute between January 2000 and June 2015, and their medical records were retrospectively reviewed. All the procedures in the present study were approved by our institutional review board (IRB number: 1508-088-695). Patients in the study were primarily diagnosed with AS, and there was no prior history of radiotherapy. Patients with AS located at any other site except the scalp were excluded from the study. The reason for such exclusion was that the scalp has a unique anatomy which significantly affects the surgical decisions. Patients with other malignancies such as hemangiopericytoma, Kaposi's sarcoma, and malignant fibrous histiocytoma were also excluded. The risk factors of demographic data of patients, horizontal and vertical dimensions of resection, and adjuvant treatments were explored, and their effects on the recurrence rates, metastasis, and patient survival were analyzed.

### 2.2. Treatment and Evaluations

Preoperative evaluation comprised pathologic confirmation of the skin biopsy specimens or reconfirmation using histologic slides at other centers, magnetic resonance imaging (MRI) of the brain, chest radiography, computed tomography (CT) of the neck, positron emission tomography (PET), and bone scan of the whole body. They all showed no evidence of metastasis to distant organs. Scalp hair was removed preoperatively, and the lesion was reevaluated. For skin margins without definitive presentation, mapping biopsies were performed in outpatient clinic to determine the extent of resection. In the operating theater, the boundary of the primary lesion was reconfirmed, and the lateral resection margins—free from the tumor—were determined. Thereafter, a wide excision was performed, while ensuring sufficient safety margins, to obtain clear lateral and deep resection margins according to the initial surgical plan (Table 1). After removing the primary lesion, an intraoperative frozen biopsy was performed to establish clear surgical margins (Figure 1). The resultant defect was reconstructed by the free latissimus dorsi (LD) muscle flap. After successful microanastomosis between the vascular pedicles of the flap (thoracodorsal (TD) artery and vein) and the recipient vessels (superficial temporal (ST) artery and vein), the raw surface was covered with the muscle flap and a split-thickness skin graft (Figure 1). Cervical lymph node dissection was performed only in patients who were suspected to have regional lymph node metastasis, as confirmed by preoperative imaging studies. Outpatient clinic-based follow-ups were performed postoperatively, every 3 months during the first year and then every 6 months over the next 1 year. During each visit, brain MRI and chest radiography were performed in each patient for determining recurrence or metastasis. At 1 month postoperatively, complete wound healing was verified, and then radiation therapy was initiated selectively based on the protocol of our institution.

### 2.3. Statistical Analysis

The Kaplan-Meier method was used to determine overall survival, median survival, and disease-free survival rates. To evaluate the association between risk factors and outcome parameters, the Cox regression test was chosen for univariate and multivariate analyses. Statistical analysis was performed using version 9.3 of the SAS program (SAS Institute Inc., Cary, North Carolina, USA). A *P* value <0.05 was considered statistically significant.

## 3. Results

We retrospectively reviewed the records of a total of 14 patients (13 males and 1 female). The patients' demographic characteristics are presented in Table 1. All patients were Korean, and the mean age at the diagnosis was 69 (range: 52–81) years, whereas the mean follow-up period was 17 (range: 8–87) months. At the time of the initial diagnosis, 9 patients had high blood pressure requiring antihypertensive medication, 1 patient had chronic obstructive pulmonary disease, 1 patient had chronic kidney disease, and 1 patient had a history of a cerebrovascular event. With regard to the postoperative adjuvant treatment, 3 patients received radiotherapy alone, 3 patients received chemotherapy alone, and 5 patients received both radiotherapy and chemotherapy. No revision surgery due to vascular compromise of the flap was required in any of these cases. Moreover, postoperative complications such as hematoma, wound infection, or flap failure were not observed. After radiation therapy was administered, partial loss of the skin graft was observed in some cases. However, the degree of loss was not significant, and wound healing was completed by secondary intention. In 1 patient, an additional split-thickness skin graft was applied to cover the raw surface in the operating room. The overall 5- and 2-year survival rates were 15% and 75%, respectively, whereas the 5- and 2-year disease-free survival rates were 7.7% and 38.7%, respectively. The mean survival duration was 32 months (Figures 2 and 3). Metastatic tumor dissemination to the lung or brain was associated with a major cause of death. Among the 14 patients, 7 patients were observed until the time of death. The major causes of death were the following: 4 cases of serious pulmonary complications as a result of lung metastasis and 2 cases of intracranial hemorrhage as a result of a metastatic brain tumor. The common chief complaints when visiting the emergency room were sudden onset dyspnea or hemoptysis in patients who had pulmonary metastasis and sudden onset altered mentality, limb weakness, or dysarthria in patients who had brain metastasis. None of the risk factors, except for a deep surgical margin for excision, were significantly associated with the rates of recurrence, metastasis, and patient survival. Although a deep excision margin was the only factor significantly associated with the rate of recurrence, it was not significantly associated with the rate of metastasis or the patient survival. The hazard ratio for local recurrence was increased to 24.15 (95% confidence interval: 2.12–275.24) when the periosteum was preserved, as compared to when the periosteum and bone were resected (*P* < 0.05) (Figure 4). Of the 14 patients, 1 experienced postoperative depression and was therefore referred to a psychiatrist.

## 4. Discussion

The poor prognosis of AS is reportedly associated with various factors. First, the definite diagnosis in these cases is often delayed or incorrect; therefore, the disease is already at an advanced stage during the initial presentation. AS usually has an insidious growth pattern, and the clinical features may vary [15, 16] (Figure 5). Benign diseases such as hemangioma or vascular malformation, pigmented skin lesions, seborrheic dermatitis or seborrheic keratosis, nodular or ulcerated skin lesions, and inflammatory skin conditions may make differential diagnosis difficult [4]. Moreover, malignant neoplasms, such as malignant melanoma, can mimic the presentation of AS [1]. These factors may often lead to the lack of recognition by patients as well as the lack of perception by physicians. Hence, a high grade of suspicion and adequate skin biopsy in the earlier stage of the disease are necessary for accurate diagnosis. Second, vascular origin of AS may be associated with poor prognosis, and AS has a high incidence of hematogenous spread [2]. The most common distant metastatic site for AS is the lung [4, 17], although the brain is also prone to the dissemination of tumor cells [17]. Third, AS tends to develop as multiple lesions, which makes it difficult to define a clear boundary for the tumor [1]. In the cases of satellite lesions, the residual tumor may be occult, even after wide excision. Fourth, cutaneous AS is a very rare disease even among malignant cancers, and the accumulated clinical experience on AS remains insufficient. Consequently, there is no clear consensus regarding the treatment protocol.

The anatomy of the scalp is unique and affects the clinical course of AS [16]. There is considerable arterial blood supply to the scalp [18]; in particular, diverse branches originating from both internal and external carotid arterial systems anastomose in the scalp. Compared to such horizontal patterns of arterial supply, venous drainage displays both horizontal and vertical patterns. The horizontal drainage of the superficial vein travels along the arterial pathway. However, there are also special vertical venous channels that are directly linked with the intracranial space. These are termed emissary veins; due to the direct interconnection of these veins, the tumor can easily spread into the brain parenchyma. This anatomic characteristic may explain higher occurrences of brain metastasis; in fact, 2 of 7 patients in the present study died due to intracranial hemorrhage after brain metastasis. Unlike the face, only a few important structures need to be preserved in the scalp, in terms of functional or aesthetic aspects. Hence, surgeons can acquire a more sufficient resection margin, free from the tumor, when performing wide excision of AS in the scalp.

After the radical resection of AS, the wide defect was reconstructed using free LD muscle flap and a split-thickness skin graft. Risk factor analysis indicated that a deep margin for excision was significantly associated with the rate of recurrence. The periosteum should be stripped off to reduce the risk of local recurrence. A wide tissue defect without any periosteum is recommended to be reconstructed using free flap transfer, and the LD muscle flap may be a good candidate regarding its size. In addition, TD vascular pedicles have compatible calibers and sufficient length as compared to ST recipient vessels. If a muscle flap is located under the skin graft, more rapid secondary healing is expected. The aesthetic outcome after reconstruction with the combination of free muscle flap and skin graft was acceptable, with considering scalp contour and skin color matching. We did not observe any complications related to the flap operation, such as hematoma under the flap, infection, or loss of the flap.

The 5-year survival rate in the present study was 15%, which is consistent with the values reported in the literature (10–50%) (Table 2) [4, 7, 11–13]. Complete excision is considered to be important for overall survival in patients with AS. However, only a few studies have described the specific surgical protocol and its relationship with prognosis. The extent of the lateral safety margin was not significantly correlated with outcome parameters, due to a small sample size. A larger number of patients in a future study may indicate a statistical association between the extent of the lateral safety margin and the clinical outcomes. The depth of excision should reach the periosteum, in order to prevent tumor recurrence.

The current primary treatment of AS involves complete excision of the tumor and adjuvant radiotherapy; however, the prognosis of AS remains obscure. We assume the mapping biopsy helps in determining surgical margin in advance, and the effectiveness of such procedure has been affirmed through previous studies in AS and extramammary Paget's disease [25, 26]. This method facilitates the detection of occult satellite lesions, and it provides indications of the more extensive resection. Aggressive excision of the tumor of the scalp may be more beneficial for patient survival. Gudewer et al. presented a case of whole scalp reconstruction with a free muscle flap and skin graft after AS resection, with a good postoperative result [1]; the aesthetic results were also satisfactory in that case. According to Lim et al. [22], radical resection with a sufficient safety margin (5 cm) may provide survival advantage. Up-to-date nonsurgical treatment modalities such as immunotherapy or gene therapy may be promising [5, 15, 20]. There are still ongoing debates about the application of chemotherapy in the standard AS treatment. Based on the current updates of literatures, chemotherapy is more recommended in case of recurring AS for the palliative purpose [2, 27–30]. We used chemotherapy ancillary to surgical resections and radiotherapy. Further research and clinical experience are necessary in order to apply new therapeutic modalities. We suggest multidisciplinary approaches to AS patient with active discussions and cooperation among physicians in different fields for maximizing the effect of treatments. For example, our institution has a sarcoma center in the cancer hospital. Medical collaborations were made among departments of plastic and reconstructive surgery, dermatology, medical oncology, radiation oncology, and neurosurgery, and feedback was exchanged before and after the surgery.

The current study had some limitations, including the retrospective study design and small sample size. Moreover, no control group was used for comparison. Hence, a future study with a larger sample size may provide more significant information.

## 5. Conclusions

AS is a rare and highly aggressive malignant tumor with a poor prognosis. We observed that only a deep margin for excision was significantly related to the rate of recurrence. Hence, ensuring the presence of a sufficient deep margin as well as an adequate lateral margin is essential during wide excision of AS. Further study is also needed to develop new treatments for AS, such as immunotherapy or gene therapy.

## Figures and Tables

**Figure 1:** Intraoperative photographs during wide excision of angiosarcoma of the scalp. A wide soft-tissue defect had been made after wide excision of the tumor (a). Reconstruction using a free latissimus dorsi muscle flap with split-thickness skin graft had been performed (b).

**Figure 2:** A Kaplan-Meier survival plot for overall survival rate. The overall 5- and 2-year survival rates were 15% and 75%, respectively.

**Figure 3:** A Kaplan-Meier survival plot for disease-free survival rate. The 5- and 2-year disease-free survival rates were 7.7% and 38.7%, respectively.

**Figure 4:** Comparison of the recurrence rates based on the status of deep resection margins. Kaplan-Meier plots stratified by the status of deep resection margins are shown. Only a deep excision margin was significantly related to the recurrence rate. The hazard ratio for local recurrence was increased to 24.15 (95% CI: 2.12–275.24) when the periosteum was preserved, as compared to when the periosteum and bone were resected (*P* value <0.05). CI: confidence interval.

**Figure 5:** Various preoperative clinical features of angiosarcoma of the scalp: ulcerative type (a), bruise-like type (b), and nodular type (c).

**Table 1:** Overall information of 14 patients with angiosarcoma of the scalp.

Patient number	Gender	Age at Dx	Tumor size at Dx (cm)	Resection margin (cm)	Deep margin	Reconstruction methods	Biopsy results	Adjuvant therapy	Profile of radiotherapy	Local recurrence (months)	Metastasis (months)	Meta area	Death (months)
1	M	52	3 × 2	1	G	FF, SG	MN	C	Null	5	69	Lung	85
2	M	70	8.5 × 5	2	B	FF, SG	MN	RT, C	63 Gy	15	21	LRR	30
3	M	61	4 × 3	3	P	FF, SG	MN	C	Null	10	12	Brain	23
4	F	64	9 × 5.5	2	P	FF, SG	MN	RT	NR	7	FL	LRR	FL
5	M	76	5 × 5	5	B	FF, SG	MN	null	Null	NE	45	Lung	48
6	M	71	5 × 4	5	P	FF, SG	MN	RT, C	61 Gy	9	13	Bone	NE
7	M	70	4 × 4	5	B	FF, SG	MN	null	Null	17	36	Brain	37
8	M	75	9.5 × 7 8.5 × 8	NR	B	FF, SG	MP	C	Null	11	FL	Null	FL
9	M	64	3 × 2.5	3	B	FF, SG	MN	RT, C	30 Gy	13	20	Lung	32
10	M	81	3 × 3	1	G	LF	MN	null	Null	7	9	Lung	13
11	M	58	3 × 3	2	P	FF, SG	MN	RT, C	61 Gy	8	10	Lung	NE
12	M	75	13 × 8	3	P	FF, SG	MN	RT, C	50 Gy	11	NE	Null	NE
13	M	81	11.5 × 6.0	3	B	FF, SG	MN	RT	42 Gy	5	NE	Null	NE
14	M	68	6 × 6	3	B	FF, SG	MN	RT	50 Gy	NE	NE	Null	NE

Dx: diagnosis; cm: centimeters; Meta area: area of metastasis; M: male; F: female; NR: not recorded; G: galea; P: periosteum; B: bone; FF: free flap; LF: local flap; SG: skin graft; MP: margin positive; MN: margin negative; RT: radiotherapy; C: chemotherapy; Gy: grays; NE: no event; FL: follow-up loss; LRR: locoregional recurrence.

**Table 2:** A review of literatures.

	Authors	Year	*N*	M (F)	Age at Dx	Race	Location of tumor	Treatment	Surgical method	Mean f/u period (months)	5-year OSR (%)	5-year DFSR (%)	2-year OSR (%)	2-year DFSR (%)	MS (months)
1	Hodgkinson et al. [12]	1979	13	7 (6)	66 (51–80)	NR	Head and neck	S (5), S + RT (5), RT (3)	NR	13 (1–96)	NR	NR	NR	NR	NR

2	Holden et al. [4]	1987	72	44 (28)	74 (56–92)	C	Scalp and face	S + RT (3), RT (69)	NR	NR (12–144)	12	NR	29	NR	15

3	Mark et al. [7]	1996	28	21 (7)	61 (6–83)	NR	Head and neck	S (12), S + CT (3), S + RT ± CT (6), RT ± CT (7)	NR	32 (3–159)	NR	26	NR	NR	NR

4	Lydiatt et al. [6]	1994	18	13 (5)	67	C (17)	Head and neck	S (6), S + RT (2), S + CT (1), CT (9)	NR	NR	33	20	NR	NR	NR

5	Morrison et al. [19]	1995	14	8 (6)	66 (49–83)	C	Scalp and face	S + RT (6), RT (3), S ± RT ± CT (11)	STSG	NR	29	NR	NR	NR	22

6	Pawlik et al. [11]	2003	29	18 (11)	71 (33–90)	C (28), A (1)	Scalp	S + RT (28), RT (1)	WE, LF (2), and STSG (26)	18.3 (3.2–106)	12	NR	NR	NR	28.4

7	Ohguri et al. [20]	2005	20	11 (9)	71 (49–91)	A (J)	Scalp	RT + IT	NR	29.5 (5–120)	NR	NR	NR	NR	36.2

8	Buschmann et al. [16]	2008	19	14 (5)	77 (59–86)	NR	Scalp	S ± RT ± CT	Oc + STSG	NR	NR	NR	NR	NR	17.2

9	Köhler et al. [21]	2008	23	11 (12)	63 (12–75)	C (19), AA (3), and A (1)	Head and neck	S + RT (19), S + CT (2), S + RT + CT (2)	WE (2 cm)	19.7 (5–108)	21.7	NR	NR	NR	NR

10	Lim et al. [22]	2010	9	5 (4)	71 (64–82)	A (K)	Scalp	S ± RT (8)	WE (5 cm) + Oc + LD + STSG + Pr + Nd	24	NR	NR	NR	100	15

11	Ogawa et al. [23]	2012	48	29 (19)	77 (58–94)	A (J)	Scalp and face	S + RT ± CT ± IT (17), S + CT + IT (2), RT ± CT ± IT (20), RT (5), and IT (4)	WE (3–5 cm)	13.7 (2.5–105.9)	NR	NR	22.1	NR	13.4

12	Dettenborn et al. [24]	2014	80	50 (30)	71 (SD 14.4)	NR	Head and neck	S (32), S + RT (38), S + CT (4), and S + RT + CT (6)	NR	55.3 (SD 74.4)	54	NR	71	NR	64.0 (CI 48.4–75.6)

13	Mullins and Hackman [5]	2015	6	5 (1)	66 (52–83)	C (4), AA (2)	Head and neck	S (1), S + RT (2), S + RT + CT (1), and C (2)	NR	42	NR	NR	NR	20	36.7 (5–76)

14	Patel et al. [14]	2015	55	39 (16)	NR	NR	Scalp and face	S ± RT ± CT (39)	NR	25.2 (4.7–227.1)	38	16	NR	NR	25.2

15	Our study	2015	14	13 (1)	69 (52–81)	A (K)	Scalp	S (3), S + RT (3), S + CT (3), and S + RT + CT (5)	WE (1–5 cm)	17 (8–87)	15	7.7	75	38.7	31 (CI 27.0–37.0)

Year: year of publication; *N*: number of patients; M: number of male patients; F: number of female patients; Dx: diagnosis; f/u: follow-up; OSR: overall survival rate; DFSR: disease-free survival rate; MS: medial survival; SD: standard deviation; NR: not recorded; C: Caucasian; AA: African American; A: Asian; K: Korean; J: Japanese; S: surgery; RT: radiation; CT: chemotherapy; IT: immunotherapy; +: and; ±: and/or; STSG: split-thickness skin graft; WE: wide excision; LF: local flap; LD: reconstruction using a free latissimus dorsi muscle flap; Oc: outer corticotomy of the calvarium; Pr: ipsilateral parotidectomy; Nd: ipsilateral neck dissection; cm: resection margin in centimeters; CI: 95% confidence interval.
